# Hydroalcoholic Extract of *Sechium edule* Fruits Attenuates QT Prolongation in High Fat Diet-Induced Hyperlipidemic Mice

**DOI:** 10.1155/2022/8682316

**Published:** 2022-07-11

**Authors:** Firdous Sayed Mohammed, Arya Ghosh, Sourav Pal, Chayan Das, Suliman Yousef Alomar, Mohsina Patwekar, Faheem Patwekar, Byong-Hun Jeon, Fahadul Islam

**Affiliations:** ^1^Department of Pharmacology, Calcutta Institute of Pharmaceutical Technology & AHS, Uluberia, Howrah 711316, West Bengal, India; ^2^Department of Pharmaceutical Sciences, Jharkhand Rai University, Ratu Rd, Kamre, Ranchi 835222, Jharkhand, India; ^3^Department of Zoology, College of Science, King Saud University, Riyadh-11451, Saudi Arabia; ^4^Luqman College of Pharmacy, Gulbarga, Karnataka, India; ^5^Department of Earth Resources & Environmental Engineering, Hanyang University, 222-Wangsimni-ro, Seongdong-gu, Seoul 04763, Republic of Korea; ^6^Department of Pharmacy, Faculty of Allied Health Sciences, Daffodil International University, Dhaka 1207, Bangladesh

## Abstract

The present study aimed to evaluate the effect of hydroalcoholic extract of *Sechium edule* (S.E.) fruits on lipid profile and electrocardiogram (ECG) parameters in high fat-diet (HFD) induced hyperlipidemic mice. In this study, grouping of animals was done as described below (*n* = 6), where group 1 is normal control, group 2 is HFD control, group 3 is HFD + atorvastatin (10 mg/kg), group 4 is HFD + S.E. extract (200 mg/kg), and group 5 is HFD + S.E. extract (400 mg/kg). The first 3 weeks animals were supplemented with HFD, and the last 3 weeks animals were supplemented with HFD along with atorvastatin (10 mg/kg) or S.E. extract (200 and 400 mg/kg). It was observed that mice of the HFD control group showed a significant rise in the total cholesterol, triglycerides, LDL-C, and VLDL-C levels and a notable decrease in HDL-C levels. In addition, a consequential increment in ECG parameters such as QT or QTc and RR interval and a noteworthy decline in the heart rate were observed in HFD control mice. Treatment with S.E. extract (200 and 400 mg/kg) showed a significant improvement in the lipid profile. Moreover, the extract also significantly normalized the prolonged QT or QTc and RR interval and the heart rate in HFD-challenged mice. Hence, we can conclude that S.E. extract encumbers the prolongation of QT or QTc and RR interval and increased the heart rate in HFD-challenged mice.

## 1. Introduction

Hyperlipidemia is a condition where an elevation of cholesterol, cholesterol esters, phospholipids, or triglycerides takes place. Hyperlipidemia is associated with atherosclerosis and other cardiovascular diseases. It is one of the most crucial risk factors which leads to coronary artery disease (CAD), which is characterized by increased cholesterol, low-density lipoprotein (LDL), and decreased level of high-density lipoprotein (HDL) in serum [1, 2]. Besides, hyperlipidemia also increased the formation of reactive oxygen species (ROS) and causes oxidative modification of LDL, which is responsible for the initiation of atherosclerosis and other associated heart diseases by an increase in inflammatory response mediated by inflammatory cytokines and activation of chemoattractant monocytes [3, 4].

Moreover, it has been stated that hyperlipidemia is one of the reasons for the advancement of cardiac arrhythmia. Cardiac arrhythmia is generally characterized by QT prolongation. Earlier studies have disclosed that a high-fat diet (HDF) promotes cardiac arrhythmic conditions and increased myocardial ischemic injury in the rat model [5]. Furthermore, many studies showed an escalation of the sensibility to atrial arrhythmia with abnormal conduction velocity in mice supplemented with HFD [6]. Also, in an *in vivo* study mice fed with HFD for 4 weeks caused abnormal electrophysiology of the heart with prolonged QT-interval [7]. Phytomedications are primarily used for wellness improvement as well as treatment of persistent, rather than life-threatening, illnesses. Conventional therapies, on the other hand, become more popular when Western medication fails to cure an illness, such as incurable cancer, novel deadly infections, and metabolic disorders [8–10].

*Sechium edule* (S.E.) is an edible plant that belongs to the family Cucurbitaceae and is also known as vegetable pear/chayote/choko/chow-chow. Mainly several amino acids are rich in fruit and seed. A lectin from the exudates of S.E. was purified. Predominantly eight flavonoids, including three C-glycosyl and five O-glycosyl flavones, were detected [11]. Substantially leaves and fruits contain some relevant characteristics such as anti-inflammatory, cardiovascular and diuretic properties. Incidentally, leaves of S.E. have been used in medicine to eradicate diseases such as hypertension and arteriosclerosis, where it also contributes to liquefy of kidney stones [12]. The immensity of fruits has been stated for the treatment of hepatoprotective [13], antiulcer [14], antiepileptic and antidepressant [15], nephroprotective [16], antidiabetic [12, 17] and antioxidant [18] activity. More to the point, recently in a streptozotocin (STZ)-induced diabetic model S.E. extract was found to reduce the level of malondialdehyde [17]. A literature survey also revealed the cardioprotective property [19] of this fruit. Additionally, it has been demonstrated that the polyphenolic extract of S.E. shoots kindle lipolysis and slows down lipogenesis in HepG2 cells [20]. Hence, based on the context that S.E. causes lipolysis and slows down lipogenesis in liver cells, the intention of the current research was to investigate the effect of hydroalcoholic extract of fruits of S.E. on HFD-induced cardiac arrhythmia in mice.

## 2. Materials and Methods

### 2.1. Plant Material

In January 2019, fruits of S.E. were collected from the market of Bangalore, Karnataka. The fruit material is taxonomically identified and authenticated at Regional Research Institute (Ay), Bangalore, where the voucher specimen is reserved for future reference under the mentioned reference number (RRCBI/MCW/7/2008).

### 2.2. Preparation of the Extract

In the first stage, the fruits were completely washed with laboratory tap water and later with distilled water. Then the fruits were chopped (thin slices) and air-dried under shade. The dried slices of fruits were freed from moisture in a hot air oven for 1 hour at 40°C. The dry and moisture-free slices of fruits were powdered using a mechanical grinder to obtain a coarse powder. For defatting, the powder was kept with a sufficient volume of petroleum ether for 72 hours. Afterward, the powder was separated and dried under shade. Then the powder was subjected to maceration with a sufficient volume of ethanol: distilled water (7 : 3) for 72 hours with intermittent shaking. Afterward, the extract was filtered and subjected to distillation to remove the solvent. The product hence obtained was reduced to a dark-colored mass by keeping in a boiling water bath for further solvent elimination. The obtained hydroalcoholic extract was preserved in a refrigerator (4°C) until further use [16, 19].

### 2.3. Drugs and Chemicals

Atorvastatin was obtained from Emcure Pharmaceuticals Ltd., India. The chemicals and diagnostic kits (total cholesterol, triglyceride, and HDL-cholesterol) were procured from Span Diagnostics, India. All other chemicals were of analytical grade. HFD pellets were obtained from Inveniolife Technology Pvt. Ltd. The diet contains 19% protein, 17.50% fat, 3.50% fiber, 3.50% ashes, vitamins, and minerals. The normal diet was also obtained from the same company which contains 16.50% protein, 8% fiber, 8% ashes, 2% fat, 1% NaCl, vitamins, and minerals.

### 2.4. Experimental Animals

Swiss albino mice (Male) weighing 25–30 g were maintained under the controlled condition of temperature (23 ± 2°C) and humidity (50 ± 5%), and a 12 h light-dark cycle was maintained. According to the guidelines, animals were housed in refined polypropylene cages with refined straw beds to facilitate easy feeding and watering. They were supplied with *ad-libitum* food and drinking water. Before the beginning of the experiment, animals were acclimatized to a laboratory environment. Experiments on the animals were carried out as per CPCSEA guidelines and the experimental protocol was approved by the Institutional Animal Ethics Committee (IAEC) (Ref. No. F4/CIPT/ADMIN/2018–19/004).

### 2.5. Acute Oral Toxicity Study

According to OECD 423 guidelines, mice were kept overnight fasting before drug administration. The animal received a single oral dose (2000 mg/kg) of S.E. extract. Following the administration of the extract, foods were retained for further 3-4 hours. Then, the animals were observed or examined once over the initial 30 minutes and intermittently for 24 hours. Besides, a special observation with care on the animals was given during the first 4 hours. The daily observation was done to identify the autonomic, central nervous system, cardiovascular, and respiratory artifacts in the animals for 2 weeks in the same circadian rhythm. Mortality (if any) was noted [21].

### 2.6. Experimental Design

This experimental work was carried out in the pharmacology laboratory of Calcutta Institute of Pharmaceutical Technology & AHS. Hyperlipidemia was induced in Swiss albino mice by feeding them with a HFD for 6 weeks [22–26]. In this experiment, after one week of acclimatization, mice were randomly divided into five groups (*n* = 6):

  Group 1: Control diet + 0.3% CMC (vehicle)
  Group 2: HFD + 0.3% CMC (vehicle)
  Group 3: HFD + Atorvastatin (10 mg/kg; p.o)
  Group 4: HFD + S.E. extract (200 mg/kg; p.o)
  Group 5: HFD + S.E. extract (400 mg/kg; p.o)

The first 3 weeks animals of all groups were treated with HFD and then the last 3 weeks animals were treated with HFD along with atorvastatin (10 mg/kg) or S.E. extract (200 and 400 mg/kg) to the respective group. After the last dose of atorvastatin or S.E. extract animals fasted for 24 hours, and then blood was drawn via retro-orbital sinus puncture for biochemical estimation. This was followed by centrifugation at 2500 rpm for 15 minutes. The obtained serum was used for the biochemical analysis.

### 2.7. Biochemical Study

The standard diagnostic kits were used for the estimation of serum total cholesterol, triglyceride, VLDL-C, and HDL-C levels. LDL-C was determined by using Friedewald equation (LDL-C = total cholesterol-HDL-C-(triglyceride/5), where (triglyceride/5) = VLDL-C).

### 2.8. Surface Electrocardiogram (ECG) Recording in Anesthetic Mice

Mice were anesthetized by intraperitoneal injection of ketamine (50 mg/kg). Standard lead II ECG metal leads were placed on different parts of the body. The negative electrode was placed on the right arm of the anesthetized mice closely about 15 mm away from the edge of the right atrium and the positive electrode was placed on the left side of the body about 20 mm below the diaphragm and ECG was recorded for 30 minutes. The ECG signals obtained from lead II were amplified and analyzed by BIOPAC (Biosystems, USA) MP36 acquisition system version 4.0 software. QT measurements and the RR intervals were used to derive the heart rate and corrected QT (QTc).

### 2.9. QT Correction

The heart rates of small rodents are several times faster than humans [25]. QT interval is highly dependent on the heart rate of the animal. Moreover, the heart rate of rodents varies extensively. The heart rate of mice is 450–500 BPM [26]. Thus, the observed QT needs to be normalized by a factor related to the heart rate for the assessment of repolarization changes. The measured QT was thus corrected using normalized Bazett's equation QTc = QT/√RR [26, 27].

### 2.10. Statistical Analysis

Results were expressed as mean ± standard error of the mean (SEM) and analyzed using one-way ANOVA (analysis of variance) followed by Tucky's multiple comparison studies where *P* value less than 0.05 was considered as significant. A component of Graph Pad Prism version 8.1 was employed for statistical analysis.

## 3. Results and Discussion

### 3.1. Acute Oral Toxicity Studies

In an acute oral toxicity study, no mortality occurred during 48 hours of observation with the selected dose of 2000 mg/kg. As the hydroalcoholic extract of S.E. fruits was found to be tolerated up to a dose level of 2000 mg/kg. For this reason, the extract was considered to be safe and a dose range of 400 mg/kg (1/5th) and 200 mg/kg (1/10th) was selected in the present study.

### 3.2. Effect of S.E. Extract on Lipid Profile

Hyperlipidemia is a notable and independent endangerment aspect of vascular complications and is recommended to cause cardiovascular obstacles through various molecular mechanisms. Analyzing the replication of injury presumption affirms that the endangerment factors such as endothelial involuntary injury, oxidation of LDL, contagion influenced transformation in endothelium to generate endothelial infirmity and a progression of cellular interactivity that terminates in atherosclerosis. The eventual clinical outcomes may include angina, myocardial infarction, arrhythmia, and sudden death [28, 29]. In the present study, it was observed that supplementation of HDF significantly increased the total cholesterol, triglycerides, LDL-C, and VLDL-C levels and decreased HDL-C levels in hyperlipidemic mice. An increase in cholesterol levels and most significantly LDL-C are the forecaster of atherosclerosis [30]. Additionally, triglycerides are in a straight line related to the progression of coronary heart diseases [31].

HFD caused a significant rise in serum total cholesterol, triglycerides, LDL-C, and VLDL-C and a decrease in HDL-C. Treatment with S.E. extract (200 and 400 mg/kg) resulted in a significant decline in total cholesterol, triglycerides, LDL-C, and VLDL-C. S.E. extract (200 and 400 mg/kg) treatment also resulted in a significant rise in the levels of HDL-C. Standard drug atorvastatin showed a more prominent effect than the extract (Table 1). Moreover, the ability of the extract to raise HDL-C was revealed in a dose-depended manner, and administration of the extract at a dose of 400 mg/kg has shown a more prominent lipid-lowering effect. Hence, the hydroalcoholic extract of the S.E. fruits has the efficiency to control the elevated lipid level.

### 3.3. Effect of S.E. Extract on ECG Parameters

It has been demonstrated that hyperlipidemia is a risk factor for the development of cardiac arrhythmia (QT-prolongation). HDF promotes QT prolongation and increased myocardial ischemic injury in an experimental model. It also causes a change in conduction velocity in the atria leading to atrial arrhythmia and QT prolongation in mice [5–7]. A prolonged QT interval has been recognized as an endangerment characteristic towards cardiovascular mortality in a diverse community, such as healthy matter [32]. The analysis of the obtained pattern of the extended QT interval is still poorly defined; the association of cardiac ion channels resembling inheritable forms and cardiac autonomic neuropathy has been proposed [33,34]. Because coronary morbidity is the most frightening thing associated with QT prolongation [32], another important powerful threat to QT elongation as a possible precedent is myocardial atherosclerotic diseases [35]. Besides, long QT is also associated with myocarditis or inflammatory heart disease, and in some cases, it causes severe prolongation of QT. This type of condition is associated with complex ventricular arrhythmia along with general ECG abnormalities [36]. In this situation, pro-inflammatory cytokines particularly (TNF*α* and IL-1*β*) increase the action potential duration by interfering with the ion channels solely involved in action potential duration and also by elevating the sympathetic drive of the heart [37]. In addition, the elongated QT interval is affiliated with different cardiometabolic threats such as hypertension, hyperglycemia, lipid disorder, obesity, and many others [38].

The present study revealed that HFD-challenged mice showed prolonged QT and RR intervals, which not only may impart ventricular arrhythmia but also be associated with increased all-cause of cardiovascular mortality. The effect of S.E. extract on ECG parameters is given in Table 2 and Figure 1. In HFD control mice there was a significant increase in QT or QTc and RR interval which indicates cardiac arrhythmia. HDF control mice also showed a notable decline in heart rate as compared with normal control mice. Treatment with S.E. extract (200 and 400 mg/kg) resulted in a significant decrease in QT or QTc and RR interval and improved the heart rate in HFD-treated mice. Hence, treatment with the S.E. extract (200 and 400 mg/kg) encumbers this QT and RR prolongation and improved the heart rate in HFD-challenged mice. These results indicate the protection of S.E. extract (200 and 400 mg/kg) against HFD-induced cardiac arrhythmia. Overall, the effect of S.E. extract on ECG parameters was in a dose-dependent manner and the administration of the extract at a dose of 400 mg/kg has shown a more prominent effect in combating cardiac arrhythmic conditions in HFD-challenged mice.

It has been confirmed that S.E. shoot extracts kindle lipolysis and inhibit lipogenesis through stimulation of the AMPK signaling pathway in HepG2 cells [20]. In this study, this mechanism may be contributed to the attenuation of hyperlipidemic conditions in HFD-challenged mice treated with hydroalcoholic extract of S.E fruits. Furthermore, this lipid-lowering ability of S.E extract probably encumbers the QT prolongation and improved the heart rate in HFD-challenged mice.

## 4. Conclusion

In the present study, it was found that the treatment with S.E. extract (200 and 400 mg/kg) notably improved the lipid profile which was indicated by a decrease in cholesterol, triglycerides, LDL-C, and VLDL-C and upgrading of HDL-C levels in HFD treated animals. Besides, the extract showed a significant cut in prolonged QT and RR intervals and also improved the heart rate. The lipid-lowering effect of the extract of S.E. fruits probably decreased the QT prolongation and RR interval and improved the heart rate in mice supplemented with HFD. Hence, the extract perks up the lipid profile and cardiac functions in HFD-challenged animals. The higher dose of the extract (400 mg/kg) showed more prominent results. The lipid-lowering effects may be due to enhancing lipolysis or inhibiting lipogenesis through stimulation of the AMPK signaling pathway. Therefore, we have to study further about the effect of the S.E. fruit extract on the AMPK signaling pathway and establish a correlation between AMPK signaling pathway inhibition and its effects on ECG.

## Figures and Tables

**Figure 1:** ECG tracing of animals of all groups. (A) Normal control showing a normal pattern of ECG with normal QT and RR intervals. (B) HFD control showing prolonged QT and RR interval. (C) HFD + Atorvastatin (10 mg/kg) showing decrease in QT and RR intervals. (D) and (E) HFD + S.E. extract (200 and 400 mg/kg) showing prominent attenuation of prolonged QT and RR interval.

**Table 1:** Effect of S.E. extract on lipid profile in HFD-induced hyperlipidemic mice.

Treatment	Total cholesterol (mg/dl)	Triglycerides (mg/dl)	HDL-C (mg/dl)	LDL-C (mg/dl)	VLDL-C (mg/dl)
Normal control	75.03 ± 1.18	73.63 ± 1.544	37.82 ± 1.01	22.48 ± 0.84	14.72 ± 0.31
HFD control	200.47 ± 3.52^###^	137.30 ± 3.02^###^	21.70 ± 0.82^###^	148.54 ± 3.03^###^	27.45 ± 0.60^###^
HFD + atorvastatin (10 mg/kg)	97.90 ± 2.50^*∗∗∗*^	85.82 ± 1.50^*∗∗∗*^	34.18 ± 0.67^*∗∗∗*^	46.55 ± 3.18^*∗∗∗*^	17.165 ± 0.30^*∗∗∗*^
HFD + S.E. extract (200 mg/kg)	103.98 ± 1.04^*∗∗∗*^	102.72 ± 1.04^*∗∗∗*^	29.22 ± 0.68^*∗∗∗*^	55.09 ± 0.97^*∗∗∗*^	20.599 ± 0.18^*∗∗∗*^
HFD + S.E. extract (400 mg/kg)	92.35 ± 2.46^*∗∗∗*^	82.55 ± 0.83^*∗∗∗*^	31.392 ± 0.43^*∗∗∗*^	44.44 ± 2.56^*∗∗∗*^	16.437 ± 0.18^*∗∗∗*^

*n* = 6, data are expressed in Mean ± SEM.^###^*P* < 0.001, HDF control vs. normal control. ^*∗∗∗*^*P* < 0.001, treatment groups vs. HDF control.

**Table 2:** Effect on S.E. extracts on ECG parameters in HFD-induced hyperlipidemic mice.

Treatment	QT interval (ms)	QTc interval (ms)	RR interval (ms)	Heart rate (bpm)
Normal control	118.24 ± 0.37	10.22 ± 0.39	133.83 ± 0.58	448.64 ± 1.85
HFD control	213.62 ± 2.10^###^	14.15 ± 0.56^###^	227.65 ± 1.16^###^	260.46 ± 1.57^###^
HFD + atorvastatin (10 mg/kg)	168.43 ± 1.16^*∗∗∗*^	12.26 ± 0.65^*∗∗∗*^	188.64 ± 1.24^*∗∗∗*^	316.04 ± 1.00^*∗∗∗*^
HFD + S.E. extract (200 mg/kg)	138.24 ± 1.02^*∗∗∗*^	10.97 ± 0.82^*∗∗∗*^	158.62 ± 1.03^*∗∗∗*^	370.30 ± 1.66^*∗∗∗*^
HFD + S.E. extract (400 mg/kg)	127.68 ± 1.32^*∗∗∗*^	10.19 ± 0.30^*∗∗∗*^	156.89 ± 0.91^*∗∗∗*^	393.15 ± 2.20^*∗∗∗*^

*n* = 6, data are expressed in Mean ± SEM.^###^*P* < 0.001, HDF control vs. normal control. ^*∗∗∗*^*P* < 0.001, treatment groups vs. HDF control.

## Data Availability

All data used to support the findings of this study are included in the article.
